The article "Dynamic Incision under Nasal Endoscope and Low-Temperature Plasma Radiofrequency Ablation for Nasal Inverted Papilloma: An Analysis of Differences in Efficacy and the Destructive Effect on Immune Function" was retracted in 2023. Reasons: signs of a paper mill; compromised peer review; unreliable results or conclusions.

# Dynamic Incision under Nasal Endoscope and Low-Temperature Plasma Radiofrequency Ablation for Nasal Inverted Papilloma: An Analysis of Differences in Efficacy and the Destructive Effect on Immune Function

**DOI:** 10.1155/2022/9618193

**Published:** 2022-10-09

**Authors:** Fang Liu, Fei Ye, Xilan Gu, Wenbin Wang, Xiaodong Yin

**Affiliations:** Department of Otolaryngology, Nanjing Medical University Hospital Affiliated Suzhou & Suzhou Municipal Hospital, Suzhou, Jiangsu 215000, China

## Abstract

**Methods:**

NIP patients (*n* = 106) admitted between January 2020 and March 2021 were selected and grouped as follows according to the random number table method: a dissection group treated with dynamical-system surgery under nasal endoscope and an ablation group treated with LTPRA. The clinical curative effects of the two procedures were compared, and the related indexes (operation time (OT), intraoperative blood loss (IBL), and length of stay (LOS)) and postoperative adverse reactions (ARs) were counted. In addition, fasting venous blood samples were collected before treatment (T0), as well as 3 (T1) and 7 days after treatment (T2) to detect inflammatory factors (IFs; C-reactive protein (CRP), interleukin-6 (IL-6), and tumor necrosis factor-*α* (TNF-*α*)) and T lymphocyte subsets (CD3+, CD4+, and CD8+). Finally, all patients received a one-year follow-up to compare the differences in prognostic survival rate and disease recurrence rate between groups.

**Results:**

The ablation group has a similar LOS to the dissection group (*P* > 0.05), but lower OT and IBL. No marked difference was observed between groups in terms of the total effective rate (*P* > 0.05), but the adverse reaction rate was higher in the dissection group compared with the ablation group (*P* < 0.05). Compared with T0, elevated CRP, IL-6, TNF-*α*, and CD3+ were observed in both cohorts at T1, with lower levels in the ablation group as compared to the dissection group, while CD4+ and CD8+ decreased in both cohorts and were higher in the ablation group (*P* < 0.05). Meanwhile, the levels of CRP, IL-6, TNF-*α*, and CD3+ in both groups were lower at T2 compared to T1, whereas those of CD4+ and CD8+ in both groups were higher at T2 compared to T1 (*P* < 0.05). As indicated by the statistics on prognostic follow-up, the two cohorts of patients showed no evident difference in the 1-year survival rate and disease recurrence rate (*P* > 0.05).

**Conclusions:**

Both dynamical-system surgery under nasal endoscope and LTPRA have good therapeutic effects on NIP, but the latter is safer and can effectively reduce the postoperative inflammatory reaction of patients and maintain the stability of immune function, which has higher clinical application value.

## 1. Introduction

Nasal inverted papilloma (NIP), one of the most common benign tumors in rhinology, is a type of papilloma that is closely related to human papilloma virus (HPV) [1]. Two epidemiological investigations have shown a higher prevalence of NIP in men than in women, affecting people aged between 6 and 89, with a predilection for middle-aged men [2]. Patients often present with nasal congestion and intranasal masses and may be accompanied by runny (sometimes bloody) nose, head and face pain, and allotriosmia [3]. At present, the cause of NIP is not clear. Most scholars believe that it is a benign true neoplasm, but it has a certain tendency of malignant transformation. Therefore, once diagnosed, it should be treated surgically for complete removal as soon as possible and terminated before the malignant transformation of the tumor [4].

Clinically, endoscopic endonasal resection, which has the advantages of less trauma and fewer postoperative complications, is often used for the treatment of NIP [5]. With the continuous development of medical technology, most scholars have tried different methods of surgical resection under nasal endoscope, among which dynamical-system surgery under nasal endoscope and endoscopic low-temperature plasma ablation (LTPRA) have achieved good results in otolaryngology and head and neck surgery [6–8]. The basic principle of LTPRA is cryoablation, which uses the energy of low-temperature plasma radio frequency to remove tissues at a low temperature (40-70 degrees), so as to maintain the safety of local mucosal structure, effectively reduce postoperative edema and pain, and shorten the recovery cycle [9]. However, there is still little clinical research about which of the two procedures is better for NIP patients.

In order to improve the therapeutic effect of NIP, this paper explores the therapeutic effect of dynamical-system surgery under nasal endoscope and endoscopic LTPRA on NIP patients and their influences on clinical curative effects, inflammatory response, and immune function, so as to provide reliable theoretical guidance for the future clinical treatment of NIP.

## 2. Materials and Methods

### 2.1. Study Area

This study was conducted in our hospital from January 2020 to May 2022.

### 2.2. Data and Methods

NIP patients (*n* = 106) including 69 males and 37 females who received treatment in our hospital between January 2020 and March 2021, were selected and randomized to the dissection group treated with dynamical-system surgery under nasal endoscope and the ablation group treated with LTPRA. 53 patients with the mean age of 47.6 were dissection group, and 53 patients with the mean age of 47.7 were ablation group. The study has obtained approval from the Hospital Ethics Committee and informed consent from all the enrolled participants.

### 2.3. Eligibility Criteria

All the participants (age>18) were diagnosed as NIP by imaging and histopathological examination in our hospital and presented no malignant transformation, with complete data and high compliance while no previous treatment, nor surgical, or drug contraindications. On the contrary, recurrent patients and those with other major diseases, immune diseases, communication disorders, surgical contraindications, serious infectious diseases, or received other drugs one week before surgery were excluded from this study.

### 2.4. Methods

Dissection group: patients were treated with dynamical-system surgery under nasal endoscope. The patient was placed in the supine position and received general anesthesia. CT localization was performed after tracheal intubation, and a German Storz nasal endoscope was placed to lock the lesion site. The lesions were then excised with an electrodynamic system under the microscope, and the scope of resection was expanded for detailed excision. After complete excision, the surgical area was washed with normal saline and sutured. Routine anti-infective treatment was performed postoperatively. Ablation group: the preoperative preparation was the same as that of the dissection group. After endoscopic placement, the LTPRA system and a disposable low-temperature plasma cutter were used to lock and completely remove the lesions, with the resection range expanded for thorough resection. The surgical area was cleaned with normal saline after the completion of the removal, followed by incision closure. Postoperative routine anti-infection treatment was also performed.

### 2.5. Outcome Measures

(1) The clinical efficacy [10] was compared. Cure referred to complete resolution of clinical symptoms, unblocked nasal cavity, epithelized and open sinus orifice, and no abnormal secretion in the nasal cavity. Marked response corresponded to basically disappeared clinical symptoms and a small amount of abnormal secretion in the nasal. Non-response was indicated if there were no improvement in symptoms and nasal secretions. Total effective rate = (marked response + cure) cases/total cases × 100%. (2) The surgery-related indicators, including operation time (OT), intraoperative blood loss (IBL), and length of stay (LOS), were counted. (3) The postoperative adverse reactions (ARs) were recorded, and the AR rate was calculated. (4) Fasting venous blood samples were collected before treatment (T0), 3 days (T1), and 7 days after treatment (T2) to determine inflammatory factors (IFs; C-reactive protein (CRP), interleukin-6 (IL-6), and tumor necrosis factor-*α* (TNF-*α*)) and T lymphocyte subsets (CD3+ and CD4+) by ELISA (R&D Systems, USA) and flow cytometry (Beckman Coulter, Hercules, CA, USA). (5) All patients received a one-year follow-up that was carried out in the form of regular review with the interval not exceeding 3 months, and the prognosis survival rate and disease recurrence rate of the two groups were recorded.

### 2.6. Statistics and Methods

The data collected were statistically processed by SPSS23.0, and differences were indicated by *P* < 0.05. The count data, denoted by percentages, were compared between groups by the chi-square test. The quantitative data are expressed by mean ± standard deviation; the data conforming to the normal distribution were tested by the *t*-test; the variance analysis and LSD post hoc test were used for comparison among groups. The survival rate was calculated and compared by the Kaplan-Meier method and the log-rank test, respectively.

## 3. Results

### 3.1. Patient Baseline Information

To ensure the accuracy of experimental comparisons between the two groups, we collected patients' baseline information for statistical analysis before the experiment. The statistical results indicated feasibility for research as there was no difference in age, gender, BMI, Krouse staging, living environment, ethnicity, and other data between the dissection group and the ablation group (*P* > 0.05, Table 1).

### 3.2. Clinical Efficacy of Two Groups

In dissection group, the cure, marked response, and nonresponse rates were 71.70%, 28.30%, and 0, respectively, with a total effective rate of 100%, while the cure, marked response, and nonresponse rates in the ablation group were 62.26%, 35.85%, and 1.89%, respectively, and the overall effective rate of 88.11%. The two groups were not statistically different in the total effective rate (*P* > 0.05, Table 2).

### 3.3. Comparison of Surgery-Related Indexes

The OT of ablation group was 72.4 ± 10.3 min, which was shorter than that of 66.5 ± 8.2 min in the dissection group (*P* < 0.05, Figure 1(a)). The IBL in the dissection group was 83.8 ± 8.2 mL, which was higher compared with the ablation group (*P* < 0.05, Figure 1(b)), while no evident difference was observed in the LOS between both dissection group and ablation group (*P* > 0.05, Figure 1(c)).

### 3.4. Incidence of Postoperative ARs in Both Groups

The bleeding rate was 5.66% in the dissection group and 1.89% in the ablation group; infection was found in 5.66% of patients in dissection group, versus none in ablation group; nasal obstruction was also higher in the dissection group versus the ablation group (3.77% vs. 1.89%); 5.66% of dissection group patients experienced epiphora while 1.89% of ablation group patients had epiphora. Taken together, the total AR rate was lower in the ablation group compared with the dissection group (*P* < 0.05, Table 3).

### 3.5. Alterations in IFs in Two Groups

Compared with CRP levels at T0, increased CRP levels were found in both cohorts at T1, with a lower level in the ablation group (7.51 ± 1.96 mg/L) compared with the dissection group. However, CRP levels in two groups were further decreased at T2 relative to T1 (*P* < 0.05, Figure 2(a)). Consistent changes were observed in IL-6 levels; IL-6 levels were increased in both groups at T1 compared to T0, and IL-6 level was 121.99 ± 20.58 pg/mL in the ablation group, which was also lower than that in the dissection group (169.96 ± 20.92 pg/mL). Meanwhile, IL-6 levels in two groups were lower at T2 compared to T1 (*P* < 0.05, Figure 2(b)). In comparison with T0, TNF-*α* level was increased at T1, with that in the ablation group was lower compared with the dissection group. However, TNF-*α* levels were declined at T2 in contrast to T1 (*P* < 0.05, Figure 2(c)).

### 3.6. Alterations in Immune Indexes in Two Groups

Compared with T0, increased CD3+ levels were observed in both groups at T1, in which the CD3+ level in the ablation group (37.18 ± 3.3%) was lower than that in the dissection group (40.45 ± 2.67%). Meanwhile, compared with T1, the CD3+ levels in both groups were reduced at T2 (*P* < 0.05, Figure 3(a)). However, CD4+ levels in the two groups were decreased significantly at T1 compared with those at T0, and CD4+ level in the ablation group was 37.00 ± 3.12%, higher than that in the dissection group. However, CD4+ levels at T2 were higher than those at T1 (*P* < 0.05, Figure 3(b)). Similarly, CD8+ levels in the two groups at T1 were lower than that at T0, but it was still higher in the ablation group than that in the dissection group. Besides, CD8+ levels at T2 were higher than those at T1 (*P* < 0.05, Figure 3(c)).

### 3.7. Prognostic Survival Rate and Disease Recurrence Rate of the Two Groups

All the subjects were successfully tracked during the prognostic follow-up. Among them, the overall mortality of ablation group was 3.77%, and that of the dissection group was 5.67%. No marked intergroup difference was found in the one-year survival (*P* > 0.05, Figure 4(a)) nor was there any statistical significance in the one-year recurrence rate between ablation group and resection group (7.55% vs. 11.32%) (*P* > 0.05, Figure 4(b)).

## 4. Discussion

The predilection sites of NIP were the ethmoid sinus, maxillary sinus, lateral wall of the nasal cavity, and frontal sinus, but because of the highly invasive nature of the disease, tumor lesions can easily invade other surrounding tissues [11]. Therefore, there will be a great risk of disease recurrence or even deterioration once the lesion is not completely removed during surgery [12]. In addition, although NIP is of epithelial origin, some studies have found abnormal bone in the tumor base, which not only elevates the potential threat of NIP but also increases the difficulty of surgical treatment [13]. It is precisely because of this that in modern clinical treatment, the surgical selection of NIP has become a focus and difficulty in clinical research. The choice of surgical approach and surgical method and how to reduce postoperative tumor residues are the key points that need to be paid attention to in the treatment of NIP.

With the continuous development and improvement of minimally invasive techniques, LTPRA has gradually become a type of minimally invasive procedure that has attracted much attention in clinical practice [14]. It works by using ions to accelerate energy harvesting and applying it to human tissue cells to ablation or solidify cells [15]. Although existing evidence has demonstrated the excellent effect of LTPRA on NIP, its specific advantages and disadvantages compared with conventional powered microdebrider are still unclear, with few research reports on this issue. Therefore, the comparison of the therapeutic effects between dynamical-system surgery under nasal endoscope and LTPRA in this paper can provide reliable reference and guidance for the selection of NIP surgical procedures in the future.

This study determined no obvious difference in clinical efficacy between dissection group and ablation group, suggesting that both procedures are ideal for the clinical treatment of NIP. However, the ablation group was observed with less OT and IBL and a lower postoperative AR rate, indicating higher safety of LTPRA than dynamical-system surgery under nasal endoscope. As we all know, without the function of coagulation, the application of traditional powered microdebrider leads to relatively more bleeding intraoperatively, which in turn interferes with the surgeon's surgical field of vision and increases the difficulty of distinguishing the tumor from the surrounding structure, resulting in reduced accuracy of operation [16]. In contrast, LTPRA, with its advantages of low-temperature operation, can quickly seal microvessels in tissues and reduce intraoperative bleeding [17]. Meanwhile, the cutter used in LTPRA has the functions of wound washing and suction device, which further ensures the clarity of the surgical field [18]. What is more, the plasma knife is flexible, which makes it easier for the surgeon to operate, and for some NIPs infiltrating into complex parts, the flexible plasma cutter is also more applicable [19]. However, a previous study mentioned that LTPRA can shorten the rehabilitation process of patients [20], which is inconsistent with our findings that there was no difference in the LOS between the two groups. This may be due to the small number of cases included in this study and the absence of severe NIP (Krouse stage IV) patients. It may also be due to the fact that both procedures are minimally invasive, so there is no significant difference in postoperative recovery time.

As far as we know, the regulation of inflammatory and immune responses is central to the survival of tumors [21]. As reported previously, inflammatory factors and immune function are closely related to NIP [22, 23]. Herein, in the intergroup comparison of the inflammatory response and immune function, it could be seen that CRP, IL-6, TNF-*α*, and CD3+ in the ablation group were lower than those in the dissection group at T1, while CD4+ and CD8+ were higher, indicating lower inflammatory response and more stable immune function of the ablation group at this time. We believe that this is because LTPRA can work at a low temperature of 40-60°C, which can reduce the thermal damage to the surrounding tissues and protect the normal structure of surrounding tissues and mucous membranes while ensuring tumor resection [24]. Moreover, the simultaneous resection and coagulation in LTPRA can also avoid the occurrence of peroxidation damage in patients, which is more conducive to maintaining the stability of patients' immune function [25]. At T0, both groups were in the initial stage after mechanical invasive surgery with obvious tissue damage, so there was no difference. On the other hand, at T1, the tissue damage tends to be basically stable, and the advantages of less tissue damage and better protection of body function of LTPRA show up at this time, resulting in a better postoperative state in patients. At T2, the injury after minimally invasive surgery has basically completed self-repair, and various functions tend to be normal, so the inflammatory factors and T lymphocyte subsets are basically consistent in both groups. Finally, this study determined no difference in the prognostic survival and recurrence between groups, which further demonstrated the ideal prognosis of NIP patients brought by the two surgical methods. But it may also be the statistical accident caused by the small number of cases mentioned above.

Thus, in the follow-up research, we will increase the number of research cases to verify the experimental findings. In addition, more surgical methods will be used as controls to investigate the clinical effects of LTPRA to further confirm its application potential. Finally, we will conduct a longer follow-up investigation on the subjects of this study to obtain more comprehensive experimental results for clinical reference.

## 5. Conclusion

Both dynamical-system surgery under nasal endoscope and LTPRA have good therapeutic effects on NIP, but the latter is safer and can effectively reduce the postoperative inflammatory reaction of patients and maintain the stability of immune function, which has higher clinical application value.

## Figures and Tables

**Figure 1:** Clinical efficacy of two groups. (a) Comparison of OT between two groups. (b) Comparison of IBL between two groups. (c) Comparison of LOS between two groups. & indicates that there is a difference compared with T0, @ indicates that there is a difference compared with T1, and # indicates that there is a difference compared with the dissection group (*P* < 0.05).

**Figure 2:** Alterations in IFs in two groups. (a) Comparison of CRP levels in the course of treatment. (b) Comparison of IL-6 levels in the course of treatment. (c) Comparison of TNF-*α* levels in the course of treatment. & indicates that there is a difference compared with T0, @ indicates that there is a difference compared with T1, and # indicates that there is a difference compared with the dissection group (*P* < 0.05).

**Figure 3:** Alterations in immune indexes in two groups. (a) Comparison of CD3+ levels in the course of treatment. (b) Comparison of CD4+ levels in the course of treatment. (c) Comparison of CD8+ levels in the course of treatment. & indicates that there is a difference compared with T0, @ indicates that there is a difference compared with T1, and # indicates that there is a difference compared with the dissection group (*P* < 0.05).

**Figure 4:** Prognostic survival rate and disease recurrence rate of the two groups. (a) The 1-year survival curve of the two groups. (b) The 1-year prognosis of disease recurrence of the two groups.

**Table 1:** Patient baseline information.

	Dissection group (*n* = 53)	Ablation group (*n* = 53)	*χ* ^2^ or *t*/*P*
Age	47.6 ± 6.0	47.7 ± 5.8	0.087/0.931
Gender			
Male	35 (66.04)	34 (64.15)	
Female	18 (33.96)	19 (35.85)	
BMI (kg/m^2^)	27.7 ± 2.3	27.8 ± 2.0	0.239/0.812
Tumor staging (Krouse)			0.448/0.799
Stage I	15 (28.30)	12 (22.64)	
Stage II	24 (45.28)	26 (49.06)	
Stage III	14 (26.42)	15 (28.30)	
Living environment			0.374/0.541
Town	33 (62.26)	36 (67.92)	
Rural	20 (37.74)	17 (32.08)	
Nationality			0.442/0.506
Han nationality	47 (88.68)	49 (92.45)	
Minority	6 (11.32)	4 (7.55)	

**Table 2:** Clinical efficacy of two groups.

Clinical efficacy	Dissection group (*n* = 53)	Ablation group (*n* = 53)	*χ* ^2^	*P*
Cure	38 (71.70)	33 (62.26)		
Marked response	15 (28.30)	19 (35.85)		
Nonresponse	0 (0.00)	1 (1.89)		
Total effective rate	100%	88.11%	1.01	0.315

**Table 3:** Incidence of postoperative ARs in both groups.

Adverse reactions	Dissection group (*n* = 53)	Ablation group (*n* = 53)	*χ* ^2^	*P*
Bleeding	3 (5.66)	1 (1.89)		
Infect	3 (5.66)	0 (0.00)		
Nasal congestion	2 (3.77)	1 (1.89)		
Epiphora	3 (5.66)	1 (1.89)		
AR rate	11 (20.75)	3 (5.66)	5.267	0.022

## Data Availability

The datasets used during the present study are available from the corresponding author request.
